# Exosomes Derived from SW480-Resistant Colon Cancer Cells Are Promote Angiogenesis via BMP-2/Smad5 Signaling Pathway

This article has been retracted.

**DOI:** 10.1155/2022/6124374

**Published:** 2022-05-19

**Authors:** Song Yang, Lei Yao, Xiaolong Wang, Hao Sun, Chaogang Du, Chengpeng Song, Jingyu Fu, Yongjun Wu, Hongwu Huang, Chuansi Wang, Yongsen Wang, Yixiang Xie

**Affiliations:** Department of General Surgery, Lu'an Hospital of Anhui Medical University, Lu'an Hospital of Anhui Province, Anhui 237005, China

## Abstract

**Background:**

Multidrug resistance is the main cause of tumor recurrence and metastasis. Therefore, it is urgent to explore the mechanism and treatment of drug resistance of tumor cells. We aim to investigate the relationship between drug resistance and angiogenesis in SW480 colon cancer cells and the possible underlying mechanism.

**Methods:**

Exosomes were extracted from SW480-sensitive or SW480-resistant colon cancer cells (SW480/oxaliplatin). The CCK-8 assay, migration assay, tube formation assay, qPCR, and Western blotting were performed in human umbilical vein endothelial cells (HUVECs). The underlying mechanisms were detected by Western blotting assays and BMP-2 si-RNA silencing assay *in vitro* and *in vivo*.

**Results:**

The conditioned medium and exosomes of SW480/oxaliplatin cells promoted proliferation, migration, and tube formation of HUVECs. The expression of BMP-2 released by SW480/oxaliplatin exosomes was 2.3-folds higher than that by SW480 exosomes. Additionally, exosomal BMP-2 inhibiting the Smad signaling pathway induced the expression of vascular endothelial growth factor and CD31. Silencing of BMP-2 partly blocks the promoting effect of SW480/oxaliplatin exosomes on angiogenesis. Moreover, SW480/oxaliplatin cells increased the BMP-2 expression, consequently promoting angiogenesis *in vivo*.

**Conclusions:**

SW480-resistant colon cancer exosomes promoted angiogenesis via the BMP-2/Smad signaling pathway, which is potential for the novel treatment for antiangiogenic therapies in colon cancer.

## 1. Introduction

Colorectal cancer (CRC) is one of the most common gastrointestinal malignancies, with the third highest incidence and the second highest mortality in all malignant tumors [1, 2]. Chemotherapy is the primary treatment for advanced metastatic tumors [3]. However, multidrug resistance (MDR) often leads to poor efficacy of chemotherapy [3, 4]. The proliferation of drug-resistant cells is accelerated and metastases to distant regions, promoting increased angiogenesis [5]. Clinically, it is often found that tumor cells have multidrug resistance to a variety of chemotherapy drugs, resulting in tumor recurrence and tumor metastasis [6, 7]. Therefore, it is of great significance to explore the mechanism and treatment of tumor-resistant cells.

Exosomes are nanoscale vesicles with a diameter of 30-100 nm secreted by a variety of living cells, which can be stable in body fluids and play the role of information transmission between cells [8]. Exosomes contain a large number of maternal-cell-derived substances, including proteins, nucleic acids, and lipids, which participate in the regulation of tumor microenvironment in the way of transmitting material information [8]. It is involved in tumor growth, invasion and metastasis, immune escape, chemotherapy resistance, and radiotherapy tolerance [9, 10]. Studies on pancreatic ductal adenocarcinoma, breast cancer, ovarian cancer, liver cancer, and lung cancer have all shown that exosome transport is involved in chemotherapy resistance [11–13]. Exosomes secreted by tumor cells and stromal cells enhanced and induced drug resistance in recipient cells by transferring their contents (DNA, mRNA, miRNA, Lnc RNA, protein, etc.) into recipient cells to alter their phenotype. However, few studies have focused on the effect of exosomes on tumor angiogenesis, especially in colon cancer.

Bone morphogenetic protein 2 (BMP-2) is a highly closed live opalics contained in the family of transgenic growth factor-*β* (TGF-*β*) [14]. The main biological function of BMP-2 is to regulate cell proliferation, chemotaxis, and apoptosis, which is closely related to the growth and development of embryos, aging, and canceration [14]. Studies have shown that BMP2 is involved in the process of apoptosis, migration, and invasion of CRC, liver cancer, gastric cancer, and lung cancer [15–17] and affects the release of immune factors by tumor cells. Feng et al. found that BMP2 was highly expressed in liver cancer tissues [18]. Overexpression of BMP2 promoted cell proliferation, migration, invasion, microvascular density, and angiogenesis and reduced cell apoptosis [18]. However, the role of BMP-2 in drug resistance and angiogenesis is not fully understood.

In this study, we investigated the relationship between drug resistance and angiogenesis in human colon cancer SW480 cells. In addition, we also determined the role of SW480 cancer cell exosomes in angiogenesis and its potential mechanism.

## 2. Methods

### 2.1. Cell Culture

SW480 colon cancer cells and SW480/oxaliplatin cells were cultured in L-15 medium containing 10% fetal bovine serum (Gibco, Grand Island, NY, USA) and 1% penicillin/streptomycin (Gibco). Conditioned medium (CM) was collected after cells were cultured in exosome-free FBS medium for 48 h. Human umbilical vein endothelial cells (HUVECs) were purchased from the cell bank of Chinese Academy of Sciences (Shanghai, China) and were cultured in RPMI 1640 medium (Gibco) containing 10% fetal bovine serum. All cells were inoculated in T25 flask and cultured in an incubator at 37°C with 5%CO2. The subculture was performed once every 2 to 3 days.

### 2.2. Exosomes Isolation

The CM was prepared for the exosome isolation. All of the following centrifugations occurred at 4°C. CM was centrifuged at 300×*g* for 10 min; 2, 000×*g* for 10 min; 10, 000×*g* for 30 min; and then at 140, 000×*g* for 90 min. After the supernatant is removed, the precipitate obtained is called exosome. The precipitation was washed and resuspended with PBS buffer and then was centrifuged again at 140 000×*g* for 90 min. Finally, the precipitates were resuspended with 100 *μ*L PBS buffer (Seyotin, China) and frozen at -80°C. The morphology of exosomes was detected by transmission electron microscopy (TEM, Hitachi, Japan).

### 2.3. Animal Experiments

The tumor was established in BALB/c nude mice. Six-week old male BALB/c nude mice were randomly divided into three groups (*n* = 6): control, SW480-exos, and SW480/oxaliplatin-exos. The mice in the control group were injected subcutaneously with SW480 cells in the groin. The mice in the SW480 group were injected subcutaneously with SW480 cells+SW480-exos in the groin. The mice in the SW480/oxaliplatin-exos group were injected with SW480 cells+ SW480/oxaliplatin-exos. After inoculation for 28 days, mice were sacrificed and acquired the tumors tissues.

### 2.4. Cell Viability Assay

The cells were collected by centrifugation and made into cell suspension at a concentration of 5-10 × 10^4^/mL. 100 *μ*L cell suspension was seeded into 96-well plates. The inoculated cell culture plates were placed in the incubator for 2 h. The culture supernatant was removed from the 96-well plate, and 100 *μ*L of medium containing different concentrations of drugs was added. After incubation for 12, 24, and 48 h, 10 *μ*L CCK8 solution (5 mg/mL) was added to each well and continued for 4 h. The 96-well plate was gently inverted to remove the supernatant. 150 *μ*L dimethyl sulfoxide was added to each well and shaken at low speed for 10 min to make the crystals fully dissolved. Finally, the value of optical density was measured at 490 nm.

### 2.5. 5-Ethynyl-2'-Deoxyuridine (EdU) Assay

EdU assay kit (RiboBio, China) was used for the measurement of cell proliferation. Cells were cultured into 96-well plates with a density of 5 × 103 for 24 hours. After the treatment of SW480-exos or SW480/oxaliplatin-exos, cells were added with EdU (50 *μ*mol/L) for 2 h. Then, cells were washed with PBS for 2 times for 5 min. 50 *μ*L 4% paraformaldehyde was added into per well for 30-min incubation at room temperature. 50 *μ*L glycine (2 mg/mL) was added and incubated in shaking table for 5 minutes. After washing with PBS again, cells were permeabilized with 0.5% TritonX-100 for 10 min. Then, cells were stained with existing Apollo dyeing reaction solution for 30 min in dark. After washing with PBS again, cells were then stained with existing Hoechest33342 for 30 min in dark to visualize the nuclei. Respective images were captured using confocal microscopy (Leica TCS SP8, Wetzlar, Germany).

### 2.6. Cell Migration Assay

Transwell Boyden chamber was used for cell migration assay. The gel was reconstructed by adding 200 microl DMEM medium to each well. Medium containing 10% FBS was added in Transwell lower chamber (600 *μ*L/well). Cell suspension (5 × 10^4) was prepared in a serum-free medium and then added into Transwell upper chamber and cultured for 24 h. After discarding the upper chamber fluid, cells were fixed with 10% neutral formaldehyde for 10 min and then stained with Giemsa for 10 min. After three times of PBS washing, three fields were randomly selected under an inverted microscope to count the number of cells.

### 2.7. Tube Formation Assay

HUVECs were planted in a six-well plate and grew to 100% fusion density (1 × 10^4). Matrigel solution was diluted to 0.05% in the medium (0.5 mg/mL). The cells were grown in medium with 0.05% Matrigel for 24 h. A similar tubular structure was observed under a microscope (×10).

### 2.8. Immunofluorescence

The prepared cell slides were soaked and washed with PBS for 3 times (5 min per time). The slides were fixed with 4% paraformaldehyde for 15 min and then soaked with PBS for 3 times. Then, cells were permeated by 0.5%Triton X-100 at room temperature for 20 min. After washing with PBS, cells were blocked with 5% goat serum for 30 min at room temperature. After washing off the blocking fluid, cells were incubated overnight with the primary antibody CD31 (Cat No.3528, Cell Signaling Technology) at 4°C. The slides were soaked and washed with PBST for three times and incubated with fluorescent secondary antibody (Cat No. FITC-60299, Proteintech, Rosemont, IL, USA) at 20-37°C for 1 h. After the nucleus is stained with DAPI (Cat No. D9542, Sigma-Aldrich, St. Louis MO, USA), images were captured using confocal microscopy (Leica).

### 2.9. RNA Extraction and Quantitative Reverse Transcriptase-PCR (qRT-PCR)

Total RNAs were extracted from cells with TRIzol Reagent (Thermo Fisher Scientific). After quantitation, RNA was reverse to cDNA using a PrimeScript RT reagent kit (Seyotin, China), and then, quantitative real-time PCR was performed by using SYBR Premix ExTaqTM II (Seyotin, China). The mRNA levels are normalized to GAPDH, and the primers used above are listed in Table 1.

### 2.10. Western Blotting Assay

The total proteins were extracted from cells or exosomes and quantified by the BCA assay kit (Seyotin, China). Proteins were separated on a 10% SDS-PAGE gel on ice and then transferred onto a PVDF membrane. After blocking with 5% bovine serum albumin (BSA), PVDF membranes were incubated with primary antibodies VEGF (Cat No.50661, CST), CD31 (Cat No.3528, CST), CD9 (Cat No.98327, CST), CD63 (Cat No.55081, CST), CD81 (Cat No.10037, CST), BMP2 (Cat No. 66383-1-Ig, Proteintech), Smad5 (Cat No. 67052-1-Ig, Proteintech), and phosphorylated Smad5 (Cat No. 9516, CST) overnight at 4°C and then goat antirabbit IgG (Cat No. 60004-1-Ig, Proteintech) at room temperature for 1 h. Bands were visualized by ECL (Seyotin, China). All antibodies used above were purchased from Cell Signaling Technology and Proteintech.

### 2.11. Small Interfering RNA (siRNA) Transfection

BMP-2 or negative control siRNA sequences were synthesized by GenePharma (Hangzhou, China). HUVECs were transfected with siRNA using Lipofectamine 2000 (Cat No. 11668019, Thermo Fisher, Waltham, MA, USA) following the manufacturer's instructions.

### 2.12. Statistical Analysis

Data were expressed as mean ± SD and analyzed for the significant difference using SPSS 22.0. The differences between two groups were analyzed by Student *t* test, and multiple groups were by one-way ANOVA. *P* less than 0.05 was considered statistically significant.

## 3. Results

### 3.1. Conditioned Medium (CM) Extracted from SW480-Resistant Colon Cancer Cells Enhance Angiogenesis

We explored the mechanisms of tumor angiogenesis by using SW480-resistant colon cancer . After culturing, the CM of both cells were collected and co-cultured with HUVECs. Compared with the CM of SW480 cells, the CM of SW480/oxaliplatin cells promoted cell activity of HUVECs (Figure 1(a)). Figures 1(b) and 1(c) find that the number of migration and tube formation of HUVECs in the SW480/oxaliplatin group was 1.64 and 1.28 times higher than that in the SW480 group. Additionally, the CM of SW480/oxaliplatin cells increased the mRAN levels and protein expression of VEGF and CD31 (markers of endothelial cell function) of HUVECs (Figures 1(d) and 1(e)). These findings suggested that the CM of SW480/oxaliplatin cells promoted the proliferation, migration, and tube formation of HUVECs.

### 3.2. Exosomes Extracted SW480/Oxaliplatin Cell Promote Angiogenesis

Based on the proven important role of exosomes in intracellular conduction, we next examined the effects of exosomes derived from the CM of SW480/oxaliplatin cell on promoting angiogenesis. After the exosomes were extracted, they were examined by TEM (Figure 2(a)). Moreover, the expression of CD9, CD63, and CD81 (exosomal positive markers) were significantly increased (Figure 2(b)). Then, the exosomes were labeled with PKH67 and co-cultured with HUVECs (Figure 2(c)).

The cell proliferation was evaluated by EdU incorporation and found that exosomes derived from the CM of SW480/oxaliplatin cell significantly enhanced proliferation of HUVECs (Figure 3). In addition, the HUVECs co-cultured with the exosomes of SW480/oxaliplatin cells had higher migration, as well as tube formation than that of HUVECs co-cultured with the exosomes of SW480 cells (Figures 4(a) and 4(b)). Furthermore, the mRAN and protein expression of VEGF and CD31of HUVECs was increased in the SW480/oxaliplatin-exos group, compared with the SW480-exos group (Figures 4(c) and S1). Collectively, we found that SW480/oxaliplatin exosomes promoted angiogenesis of HUVECs.

### 3.3. BMP-2 Increased in SW480/Oxaliplatin Exosomes and Enhanced Angiogenesis via Inhibiting the Smad Signaling Pathway

Next, we investigated the potential mechanisms by which SW480/oxaliplatin exosomes promote angiogenesis. As displayed in Figure 4(c), compared with SW480 exosomes, SW480/oxaliplatin exosomes decrease the expression of phosphorylation Smad5 in HUVECs. Previous studies report that BMP-2 is a member of transforming growth factor- *β*/BMP superfamily, which exerts a variety of biological functions by regulating TGF-*β*/Smad signaling pathways [12]. The results of Western blotting showed that the expression of BMP-2 in SW480/oxaliplatin exosomes was 2.3-folds higher than that in SW480 exosomes (Figure 5(a)). To confirm the importance of BMP2 in SW480/oxaliplatin exosomes promoted angiogenesis, we performed siRNA-mediated knockdown in HUVECs. As shown in Figures 5(b) and 5(c) and S2, knockdown of BMP2 attenuates the increasing effect of SW480/oxaliplatin exosomes on cell proliferation, migration, and tube formation. Moreover, immunofluorescence and Western blotting indicated that silencing of BMP2 significantly reduced the expression of CD31, VEGF, and phosphorylation Smad5 induced by SW480/oxaliplatin exosomes (Figures 5(d) and 5(e)). Collectively, high levels of BMP-2 contained in SW480/oxaliplatin exosomes inhibited the Smad signaling pathway, thus promoting angiogenesis of HUVECs.

### 3.4. SW480/Oxaliplatin Exosomes Promote Angiogenesis *In Vivo*

Next, we investigated the proliferation and angiogenesis of SW480/oxaliplatin exosomes in mice. After the injection for 28 days, mice in the SW480/oxaliplatin group had bigger size and tumor volumes than that in the SW480 group, and there was significant difference between the two groups (*P* < 0.05, Figures 6(a) and 6(b)). Moreover, more BMP2-positive cells were observed in mice of the SW480/oxaliplatin group than SW480 group (Figure 6(c)). Then, we detected the angiogenesis of SW480/oxaliplatin exosomes *in vivo* by immunofluorescence staining of CD31. Compared with the SW480 group, more CD31-positive cells were found in the SW480/oxaliplatin group (Figure S3). The results of Western blotting showed the up-regulation of VEGF and CD31 protein expression in the SW480/oxaliplatin group (Figure 6(e)). These results indicated that SW480/oxaliplatin exosomes could enhance proliferation and angiogenesis *in vivo*, which could via the up-regulation of BMP2.

## 4. Discussion

Multidrug resistance refers to the simultaneous resistance of tumor cells to various drugs with different structures and chemotherapy mechanisms [4]. Mechanisms of drug resistance have been reported, including (1) activation of the drug target enzyme DNA topoisomerase N or detoxifying enzyme glutathione S-transferase [19]; (2) DNA self-repair [20]; and (3) apoptosis resistance of cancer cells and changes in some signaling pathways [21]. ATP-binding cassette (ABC) is one of the main causes of multidrug resistance of tumor cells, which can extract drugs from tumor cells to the outside of the cell through ATP-dependent membrane transporter to reduce the concentration of drugs in the cell [22]. However, how drug-resistant cancer cells regulate angiogenesis remains unclear. In this study, we found that exosomes derived from SW480/oxaliplatin cells promoted cell proliferation and migration and ultimately angiogenesis. The high levels of BMP-2 contained in SW480/oxaliplatin exosomes promote angiogenesis by inhibiting the Smad signaling pathway.

Previous studies considered exosomes to be merely “fragments” of exogenous cells. An increasing number of studies have found that exosomes play an increasingly important role in mediating cell-to-cell communication [23, 24]. It can be taken up by the recipient cells by carrying a variety of molecules including proteins, miRNA, DNA, and lipids and play a series of biological roles in the recipient cells [24]. Tumor cell-derived or tumor-associated exosomes are closely related to the formation of tumor drug resistance [25]. Adriamycin-resistant breast cancer cell line MCF-7/ADR can mediate the formation of drug resistance of sensitive cells MCF-7 through exosomes [26]. Cancer-associated fibroblasts (CAFs) secreted exosomes and promote metastasis and chemotherapy resistance of CRC [27]. The main mechanisms of exosomes mediating the formation of tumor drug resistance are as follows [28, 29]: (1) exosomes carrying drugs out of the body; (2) exosomes delivering drug-resistant proteins, which are one of the main mechanisms mediating the formation of tumor drug resistance; and(3) exosomes delivering noncoding RNAs (ncRNAs). In this study, we found that the proliferation, migration, and catheterization of HUVECs co-cultured with SW480/oxaliplatin exosomes were enhanced, suggesting that exosomes of drug-resistant cells could increase the angiogenesis of endothelial cells. It will be of great theoretical and practical significance to identify specific biomolecules that affect vascular production in exosomes of drug-resistant cells.

BMP2 mRNA expression has been found in breast cancer, and it has been shown that BMP2 promoted the proliferation of MCF-7 cells [30]. Hardwick et al. detected the expression of BMP-2 in colon tissue of 6 types of colon cancer and genetic adenomatous polyposis (FAP) patients and concluded that BMP-2 resulted in decreased apoptosis and cell adhesion in mature colon epithelial cells [31]. Sporadic early-onset colorectal cancer (EOCRC) has increased expression of BMP2, which is different from APC-mutated organs [32]. Smad4-deficient CRC cells induce high levels of BMP2 in fibroblasts, which enhance CRC invasiveness and metastasis [33]. Our study demonstrated that secretory BMP-2 acts as a tumor promoter by promoting angiogenesis in the tumor microenvironment. In addition, TGF-*β* inhibited BMP2 mRNA expression in primary embryonic rats or osteocyte cultures [34]. Consistent with this, we found TGF*β*1 attenuated the enhanced angiogenesis caused by SW480/oxaliplatin exosomes in HUVECs.

Smad5 is a TGF-*β* superfamily protein that transmits signals from the cell membrane to the cell nucleus via the TGF-*β* signaling pathway [35]. When Smad5 is degraded or deleted, normal signaling is disrupted, allowing cells to escape TGF-*β*-regulated growth inhibition and becomes cancerous [35]. The down-regulation of Smad5 inhibited the expression of N-cadherin, matrix metallopeptidase 9, Snail, and Vimentin while elevating E-cadherin expression, thus inhibiting EMT, cell proliferation, migration, and invasion in NPC [36]. Through the interaction between TGF/Smad pathway and Wnt pathway, the TGF/Smad pathway can jointly coordinate the occurrence of tumor epithelial to mesenchymal transition (EMT) [37]. After the occurrence of tumor EMT, the expression of N-mucin is increased. It weakens the adhesion between tumor cells, facilitates metastasis and infiltration, and promotes the movement and metastasis of tumor cells [38]. BMP-2 plays a different role in different stages of tumor progression by acting on the Smad signaling pathway. BMP-2 promotes epithelial-to-mesenchymal transition and breast cancer stemness via Rb and CD44-Smad4 signaling pathways [39]. The proliferation of ovarian cancer cell lines was enhanced by BMP2 and suppressed by dorsomorphin via Smad5 in vitro [38]. BMP/Smad5 signaling plays an important role and, therefore, becomes a potential therapeutic target in serous ovarian cancer.

## 5. Conclusion

In summary, our results suggested that BMP-2-rich exosomes inhibited the Smad signaling pathway, thereby promoting angiogenesis and cell drug resistance. Our findings would provide new insights into the potential of BMP-2 as a novel antiangiogenesis target in CRC.

## Figures and Tables

**Figure 1:** Conditioned medium (CM) extracted from SW480-resistant colon cancer cells enhance angiogenesis. HUVECs treated with CM of SW480/oxaliplatin and SW480 cells. (a) Proliferation assay of HUVECs. (b) The Transwell assay determined the HUVECs migration. (c) Photomicrographs of tube-like structures and quantification of the tube number. (d) The mRNA level of VEGF and CD31. (e) Then, protein expression of CD31 and VEGF in HUVECs. All above experiments were repeatedly performed 3 times; data are shown as the means ± SD. ∗*P* < 0.05, ∗∗*P* < 0.01.

**Figure 2:** Characterization of exosomes of SW480/oxaliplatin cells. Exosomes were extracted from SW480/oxaliplatin and SW480 cells and then co-cultured with HUVECs. (a) Transmission electron photomicrograph of exosomes. (b) Protein expression of CD9, CD63, and CD81. (c) Confocal images of PKH67-labeled exosomes taken up by HUVECs. All the above experiments were repeatedly performed 3 times; data are shown as the means ± SD. ∗*P* < 0.05, ∗∗*P* < 0.01.

**Figure 3:** SW480/oxaliplatin cell-derived exosomes promotes cell proliferation. Exosomes were extracted from SW480/oxaliplatin and SW480 cells and then co-cultured with HUVECs. Effects of SW480/oxaliplatin cell-derived exosomes on proliferation of HUVECs were detected by EdU. All the above experiments were repeatedly performed 3 times; data are shown as the means ± SD. ∗*P* < 0.05, ∗∗*P* < 0.01.

**Figure 4:** SW480/oxaliplatin cell-derived exosomes accelerates angiogenesis. Exosomes were extracted from SW480/oxaliplatin and SW480 cells and then co-cultured with HUVECs. (a) The Transwell assay determined the HUVECs migration. (b) Photomicrographs of tube-like structures and quantification of the tube number. (c) The protein expression of CD31, VEGF, and phosphorylation Smad5 in HUVECs. All the above experiments were repeatedly performed 3 times; data are shown as the means ± SD. ∗*P* < 0.05, ∗∗*P* < 0.01.

**Figure 5:** SW480/oxaliplatin exosomes are enriched in BMP-2, which improve angiogenesis via the inhibition of the Smad signaling pathway. HUVECs were co-cultured with SW480/oxaliplatin exosomes (40 *μ*g/mL) with or without the treatment of si-RNA. (a) The expression of BMP-2 in exosomes. (b) Proliferation assay of HUVECs. (c) The Transwell assay determined the HUVECs migration. (d) The expression of CD31 detected by immunofluorescence. (e) The protein expression of VEGF and phosphorylation Smad5 in HUVECs. All above experiments were repeatedly performed 3 times; data are shown as the means ± SD. ∗*P* < 0.05, ∗∗*P* < 0.01.

**Figure 6:** SW480/oxaliplatin exosomes promotes angiogenesis in vivo. BALB/c nude mice were injected with SW480 cells and SW480-exos or SW480/oxaliplatin-exos for 28 days (*n* = 6). (a and b) The size and volume of the subcutaneous tumors in mice. (c) BMP-2 expression detected by immunohistochemical staining. (d) The protein expression of VEGF and CD31 in tumors. All above experiments were repeatedly performed 3 times; data are shown as the means ± SD. ∗*P* < 0.05, ∗∗*P* < 0.01.

**Table 1:** Primer sequences used for qRT-PCR.

Genes	Primer Sequences (5'→3')
CD31	F: AACAGTGTTGACATGAAGAGCC
	R: TGTAAAACAGCACGTCATCCTT
VEGF	F: GCACATAGAGAGAATGAGCTTCC
	R: CTCCGCTCTGAACAAGGCT
*β*-actin	F: CGTAAAGACCTCTATGCCAACA
	R: CGGACTCATCGTACTCCTGCT

## Data Availability

The data used to support the findings of this study are available from the corresponding author upon request.

## Supplementary Materials

Supplementary Materials Figure S1 SW480/oxaliplatin cell-derived exosomes promote angiogenesis. The mRNA expression of CD31 and VEGF. Data are shown as the means ± SD. ∗*P* < 0.05, ∗∗*P* < 0.01. Figure S2 SW480/oxaliplatin exosomes improve cell proliferation. The Transwell assay determined the HUVECs migration. Data are shown as the means ± SD. ∗*P* < 0.05, ∗∗*P* < 0.01. Figure S3 SW480/oxaliplatin exosomes promotes angiogenesis *in vivo*. The expression of CD31 detected by immunofluorescence. Data are shown as the means ± SD. ∗*P* < 0.05, ∗∗*P* < 0.01.
